The article "A Description of Handgrip Strength in the Very Older Adult People Living in Rural Vietnam and Its Association with Daily Functions" was published in 2021. Journal: Biomed Res Int.

# A Description of Handgrip Strength in the Very Older Adult People Living in Rural Vietnam and Its Association with Daily Functions

**DOI:** 10.1155/2021/1237547

**Published:** 2021-07-08

**Authors:** Nga Thi Thuy Nguyen, Thanh Xuan Nguyen, Anh Trung Nguyen, Thu Thi Hoai Nguyen, Tam Ngoc Nguyen, Huong Thi Thu Nguyen, Huong Thi Thanh Nguyen, Thang Pham, Huyen Thi Thanh Vu

**Affiliations:** ^1^Hanoi Medical University, Hanoi 100000, Vietnam; ^2^National Geriatric Hospital, Hanoi 100000, Vietnam; ^3^Dinh Tien Hoang Institute of Medicine, Hanoi 100000, Vietnam

## Abstract

**Objective:**

To describe handgrip strength (HGS) and identify associated factors in community-dwelling older adults in rural Vietnam.

**Methods:**

A cross-sectional study was conducted in community-dwelling older adults 80 years and over in five rural communities in Hanoi, Vietnam. Age-gender-BMI stratified HGS values were reported as means and standard deviations. Demographic characteristics, malnutrition, risk of fall, basic activities of daily living (ADL), and instrumental activities of daily living (IADL) were investigated. Multivariate linear regression explored the association between HGS and these factors.

**Results:**

In 308 participants, mean age was 85.4 ± 4.2 years. Mean HGS was 21.6 ± 6.1 kg for males and 15.3 ± 4.3 kg for females. HGS in our sample was generally lower than that in other European countries and Asian threshold. Low HGS was correlated with older age (*β* = −0.196, *p* < 0.001), female (*β* = −0.443, *p* < 0.001), low education (*β* = −0.130, *p* < 0.05), risk of falls (*β* = −0.114, *p* < 0.05), and lower IADL (*β* = 0.153, *p* = 0.001).

**Conclusions:**

The age-gender-BMI stratified HGS values of 80 years and over community-dwellers in rural Vietnam were described. HGS decreased with advanced age, female, low education, high risk of falls, and impaired IADLs. The results could provide useful reference data for further investigations and measures in clinical practice.

## 1. Background

Handgrip strength (HGS) is an indicator of muscle strength primarily generated by the flexor muscles of the hand and the forearm and measured by using dynamometers. Low HGS in older adults is primarily explained by the aging process as neural and muscular decline accompanied by physical inactivity and malnutrition. Impairment in HGS below a clinically relevant threshold results in difficulties in performing common daily activities [1] and mobility [2] and affects independence in basic daily life activities. Given its good predictive accuracy and simplicity, HGS can serve as early detection for the health conditions of older adults in a community to avoid or slow down negative outcomes by applying appropriate preventive and therapeutic interventions [3].

Over the past decade, HGS has been measured in many countries, and normative reference data stratified by gender and age is used in clinical practice [4]. Almost all researches on handgrip strength have exclusively been conducted in western societies where an affluent and sedentary lifestyle is omnipresent [5]. In Asian countries, Malhotra et al. [6] assessed HGS and related sociodemographic factors in Singapore, and Yu et al. [7] updated the Chinese reference values of HGS in 2017. Since the HGS value shows a great variation across regions and countries, reference data of locally specific areas is of value. However, published studies investigating HGS reference data and possible associated factors in the Vietnamese population have been limited. The recent study showed the prevalence of low HGS (24.9%) as part of frailty definition in Vietnam [8] in older hospitalized patients; hence, the data might be insufficient as the reference values for the Vietnamese older adult population.

Vietnam is a typical developing country in Southeast Asia having a high rate of the aging population. In 2009, the percentage of people aged 60 or over was 8.7% and will estimate an increase of up to 26.1% in 2049 [9] raising the demand for caring. The Vietnamese government is committed to promoting active and healthy aging to maximize older adults' physical, social, and mental well-being in order to promote living independence and reduce the burden on family members. Independent living is an important indicator of active aging; however, almost all older people 80 years old and over who have significant muscle weakness seek private support due to limitations in activity of daily living [10]. These elderly could have a better awareness of the importance of muscle strength and are thus willing to engage more in interventions preserving muscle to promote health and independence in older age. The present study is aimed at describing HGS and identifying its association with daily functions in people aged over 80 years living in rural Vietnam.

## 2. Methods

### 2.1. Study Design and Participants

A cross-sectional study was conducted to recruit eligible participants between September and October 2015 in five rural communities of Hanoi, Vietnam. We included community-dwelling subjects aged ≥80 years participating in the examination in a commune health center. Older adults who were unable to answer questionnaires and follow instructions were not included. The sample size was calculated by G-power software with a confidence level of 0.05 and 90% power (*β* = 0.10) in a two-tailed test that determines effect sizes of 0.61 (0.45–0.83) indicating odds ratio between sarcopenia and IADLs [11] and 10% attrition rate. The sample size calculation indicated that at least 306 subjects were needed. In this study, 308 participants were included.

### 2.2. Data Collection

After identifying eligible participants, the study was verbally explained to participants, and they were asked for oral informed consent. Each participant next received a face-to-face interview to fill in the questionnaires and completed the examinations comprising HGS measurements and Timed Up and Go Test by trained researchers. The study was approved by the National Geriatric Hospital Research Ethics Committee, Hanoi, Vietnam, with the reference number: 1337/IRB-NGH.

### 2.3. Measures

#### 2.3.1. HGS Measurement

Handgrip strength was measured by a dynamometer (Jamar™ Hydraulic Hand Dynamometer 5030 J1, USA). Participants were asked to sit on a chair, bend the elbow at a 90-degree angle, and not touch the body. The participants gripped the dynamometer as hard as possible with each hand. Measurements were taken a total of four times, two times in each hand, alternating between hands. The highest of the four grip measurements was used to be maximum grip strength (kilogram). The calibration accuracy was checked on the machine to ensure reliable and accurate results of muscle strength.

#### 2.3.2. Demographic Characteristics

Demographic information about age, gender, marital status, educational level, number of current medications, and lifestyle of currently consuming alcohol and smoking was obtained using a standardized self-reported questionnaire. Height and weight are measured with the participants wearing light clothing and no shoes, using a fixed stadiometer and a digital scale, and used to compute body mass index (BMI). BMI was divided into 3 groups as underweight (BMI < 18.5), normal weight (18–23), and overweight (>23) [12].

#### 2.3.3. Geriatric Conditions

The risk of fall was assessed by the Timed Up and Go Test (TUG) [13]. The TUG was measured the time participants stood up out of the chair, walked 3 m, turned around, walked back to the chair, and sat down. Participants were defined as having the risk of fall if they had TUG > 12 seconds. The instrumental activities of daily living scale (IADLs) was used to assess independent living skills necessary to live in the community. There are 8 domains of function measured with the Lawton IADL scale: meal preparation, nursing and personal care, homemaker services, financial and medication management, and/or continuous supervision. A summary score ranges from 0 (low function, totally dependent) to 8 (high function, totally independent) [14].

Activities of daily living (ADL) was used to assess functional status as a measurement of the participant's ability to perform activities of daily living independently. The scale assesses six functions of bathing, dressing, toileting, transferring, continence, and feeding. A score of 6 indicates full function and 0 indicates total dependence.

The presence of malnutrition was determined by 10-item Nutrition Screening Initiative (NSI) [15]. Nutrition scores were categorized by NSI criteria for >6 points as high, 3-5 points as moderate, and 0-2 points as low risk of malnutrition.

### 2.4. Statistical Analysis

Analysis of the data was performed using SPSS version 20.0 (IBM Corp., Armonk, NY, USA). Continuous variables were presented as means ± standard deviation, and categorical variables were presented as frequencies and percentages. Group comparison of quantitative parameters with normal distribution was analyzed using the *t*-test/ANOVA to examine the association between HGS and demographic characteristics, risk of falls, and nutritional status. Pearson correlation was used to examine the association of HGS and IADLs score and ADL score.

HGS were presented as means ± standard deviation and stratified by age (80-84 years, 85-89 years, 90-94 years, and 95 years and older), gender, and BMI (<18.5, 18.5-23.0, and >23.0). Multiple linear regression analyses were used to explore the association between HGS and demographic characteristics, risk of falls, cognitive function, and nutritional status. HGS was included as a dependent variable. The independent variables which had a *p* value ≤ 0.2 on univariate analysis were included in the model. Statistical significance was defined as any *p* value of <0.05.

## 3. Results

A total of 308 participants were included in this study, with a mean age of 85.4 ± 4.2 years old, which ranged from 81 years old to 106 years old. Female was accounted for 64.6%. The HGS value decreased with age and female group and was significantly lower in the advanced age. Participants who had higher education levels (secondary/high school or higher) and who were married showed higher HGS. There was a significantly decreased HGS in participants having high risk of fall (*F* = 19.649, *p* < 0.001) and lower IADL score (*r* = 0.263, *p* < 0.001) (Table 1).

Table 2 shows the means and standard deviation of HGS by age group, gender, and BMI. Generally, the mean HGS found in this study among males was 21.6 (6.1) kg and among females 15.3 (4.3) kg. The youngest age group (80-84 years old) had a higher HGS value in both male and female groups compared to others, while it was much lower especially for females in the oldest age group (90+ years old). The mean HGS showed remarkably lower in females and a decreasing trend with increasing age among all three BMI groups in both genders (Table 2).

As a result of multiple linear regression analyses showed in Table 3, the HGS was decreased with advanced age, female, illiterate, risk of fall, and low IADLs score. The older participants tend to have lower HGS, where the progression in age by one year corresponds to a reduction of HGS by 0.270 kg. There was an average reduction of 5.361 kg in the grip strength of females relative to males (*β* = −0.443, *p* < 0.001). In addition, people who are illiterate correspond to a decrease by 1.58 kg in HGS (*β* = −0.130, *p* < 0.05). The risk of fall was associated with lower HGS (*β* = −0.114, *p* < 0.05), with a decrease of 1.328 kg in the grip strength compared to those without risk of fall. The IADL score was positively correlated with HGS (*β* = 0.153, *p* = 0.001), which means that each score of IADLs was expected an increase by 0.595 kg in the HGS.

## 4. Discussion

This study is aimed at investigating HGS value stratified by age, gender, and BMI in very old Vietnamese older adults and identifying the association with daily functions. The mean HGS found in this study among men was 21.6 kg and among females 15.3 kg, which was generally lower than the threshold according to the consensus of the Asian Working Group for Sarcopenia in 2019 (28.0 and 18.0 kg for male and female, respectively) [16]. For the first time, the HGS values for 80 years old and over of the Vietnamese population are presented, providing reference values for screening tests. Because of the severity of consequences of age-associated muscle weakness in very old people, age-gender-BMI-specific HGS helps to identify individuals with low muscle strength and to plan specific preventive health strategies to increase functional independence and quality of life.

In our study, we examined the very old population; therefore, HGS could be expected to be lower than the threshold. However, compared to HGS of the Swiss sample (80 years and over) which reached around 28 kg for male and 19 kg for female, the older people in our study presented with a lower strength value in both men and female [17]. Although the values for grip strength obtained were generally lower than reference values of Western counterparts [18], it was similar to those reported in 80 years old and over Singaporean (20.5-22.9 kg in men and 12.0-13.7 kg in women) in a comparative study [6]. Other than genetic and environmental factors that may influence the country-specific differences in HGS, in Vietnam, 72.9% of the elderly live in rural areas with disadvantaged living conditions [19]. They tend to have a low education level [20]; risky behaviors such as physical inactivity, smoking, and drinking [21]; and malnutrition across the lifespan [22]. Besides, 70% of rural older adults in Vietnam suffered from noncommunicable diseases, especially cardiovascular diseases, diabetes, kidney diseases, and cancer [23]. Those factors might contribute to low HGS in this rural population. The reference values for older people aged 80 and over in Vietnam help to identify older people with low HGS, an additional reference for the old and oldest groups, and to establish specific strategies to lower the risk of adverse outcomes.

HGS was declined gradually with age and was higher in men than females, which is consistent with other studies [24]. The aging process causes degenerative changes, and reduction of muscle mass makes HGS reduced over the lifetime, especially in females who have less muscle fibers than males [25]. This study also found that the higher education levels were associated with higher HGS which was consistent with previous Korean studies [26]. Education also provides basic knowledge and life skills to get better access to information and resources to promote health during the whole lifespan [27]. The association could be driven by lower social position and reduced access to resources of those with low education in rural areas. In addition, the higher the educational level, the more conscious of physical activity and diet in maintaining health which may also affect HGS [28]. Therefore, it is possible that the awareness of exercises or dietary patterns according to the education level is eventually related to HGS. In Vietnam, the participants had limited opportunities for high education in their years; current lower educated older people should be provided with appropriate education and information about optimal nutrition and exercise.

Low HGS was associated with a higher risk of falls. Similarly, research in Taiwanese community-dwelling older adults has claimed HGS as an independent factor of one-year fall episode and recommended HGS as the most feasible measure rather than other functional tests [29]. Approximately 30% of the community-dwelling older adults, aged 65 years and over, fall at least once per year, and about 15% fall two or more times per year which causes serious adverse events [30]. Our result also highlighted a very high rate of older adults who had a risk of falling in 80 years and over living in the community in Vietnam. Screening HGS in terms of large-scale community settings would be recommended for identifying the risk of future falls and even fractures to apply interventions to avoid the spiral of negative outcomes.

After controlling for other variables, HGS was significantly associated with IADL disability, but not ADL disability. Similar to our finding, HGS was demonstrated as a predictor of IADL disability in 65+-year-old Japanese community-dwelling older adults [31]. Impairment in HGS results in difficulties in performing common daily activities in the community like shopping, preparing meals, transportation, and housekeeping which are closely related to hand flexibility. Loss of independence demands more caregiver support and negatively affects social interaction, wellbeing, and overall quality of life [32]. The very old community-dwelling adults exhibited a poor performance in all IADLs which emphasized the urgent of interventions to improve muscle strength to prevent an accelerated decline in IADLs disability. Our finding suggests that preserving HGS is likely to promote independent living that increases opportunities to participate in active aging for this vulnerable population. In addition, early detection of low HGS might provide an insight into current IADLs function and indicate future demand for supporting and caring in the Vietnamese oldest population.

To prevent falls and increase life independence in older adults, our study has an important clinical implication. Planning community healthcare programs for people of advanced age should consider HGS as a crucial factor. It is essential for a specialized muscle training program that considers the special characteristics of older people in their 80s. However, our present study also had some limitations. As this study has a cross-sectional design, a causal effect association could not be established. Furthermore, this study recruited people from rural rather than urban areas; the results may be limited to generalize to all older adults of our multiethnic country. We also highlight as a limitation of the convenience sample method composed of older adults who were able to go to the healthcare center, which possibly contributed to the noninclusion of individuals with reduced handgrip strength and ADL disability. It is suggested that a study conducted with older seniors should include home visits as a strategy for data collection, to cover those with lower functional performance.

## 5. Conclusion

This study revealed the age-gender-BMI stratified reference data of HGS in 80 years and over community-dwelling older adults in rural areas in Vietnam. Our result indicated the low values of HGS observed in this population compared to other European countries and Asian threshold. The association between HGS and age, gender, education level, risk of fall, and IADLs was found statistically significant. These results could provide useful reference data for further investigations and measures in clinical practice, as its simple, time-efficient, and noninvasive method of measuring HGS is especially useful to identify vulnerable older adults and promote independent living in the community setting.

## Figures and Tables

**Table 1:** Characteristics of the study's participants according to measurement of handgrip strength.

	Total, *n* (%)	HGS mean (SD)	95% CI	*F*/*r*	*p* value
Age					
*80-84*	152 (49.4%)	18.4 (6.2)	17.5-19.4	7.347	0.001
*85-89*	109 (35.4%)	16.8 (5.2)	15.8-17.8		
*≥90*	37 (12.0%)	15.0 (5.0)	13.5–16.5		

Gender					
*Male*	109 (35.4%)	21.6 (6.1)	20.5–22.8	25.204	<0.001
*Female*	199 (64.6%)	15.3 (4.3)	14.7–15.9		

Education					
*Illiterate*	108 (35.1%)	14.8 (4.1)	14.0–15.6	29.348	
*Primary school*	169 (54.9%)	17.7 (5.6)	16.8-18.5		
*Secondary school*	23 (7.5%)	24.1 (5.5)	21.8-26.4		<0.001
*High school and higher*	8 (2.6%)	25.5 (5.7)	16.7–18.0		

Marital status					
*Single*	13 (4.2%)	15.4 (5.8)	11.9–19.0		
*Married*	191 (62.0%)	18.5 (6.1)	17.7–19.4	11.114	<0.001
*Widowed/widower*	104 (33.7%)	15.4 (4.5)	14.5–16.3		

BMI					
*<18.5*	88 (28.6%)	17.1 (5.5)	15.9–18.2	1.035	
*18.5-23*	166 (53.9%)	17.1 (5.7)	16.3–18.1		0.356
*>23*	54 (17.5%)	18.4 (6.0)	16.6–20.2		

Malnutrition					
*Low risk*	121 (39.3%)	18.2 (6.1)	17.1–19.2	1.767	
*Moderate risk*	48 (15.6%)	17.0 (5.2)	15.5–18.5		0.173
*High risk*	139 (45.1%)	16.8 (5.6)	15.9–17.7		

Risk of fall (TUG score)					
*No*	171 (55.5%)	18.6 (5.8)	17.7–19.5	19.649	<0.001
*Yes*	137 (44.5%)	15.8 (5.4)	14.8–16.7		

Number of current medications (mean (SD))	0.4 (0.6)	17.5 (5.9)	16.9–18.2	0.087	0.128^∗^

ADL score (mean (SD))	4.5 (2.6)	17.5 (5.9)	16.9–18.2	0.088	0.123^∗^

IADL score (mean (SD))	5.9 (0.4)	17.5 (5.9)	16.9–18.2	0.263	<0.001^∗^

*p* value by ANOVA/independent *t*-test; ^∗^using Pearson correlation. Activities of daily living (ADL) score (range 0–6, a higher number indicate higher independence). Instrumental activities of daily living scale (IADLs) score (range 0-8, a higher number indicate higher independence).

**Table 2:** Means and standard deviations (SD) of handgrip strength (kg) stratified by gender, sex, and BMI.

Age	Females					Males				
	*n*	Total	Underweight	Normal weight	Overweight	*n*	Total	Underweight	Normal weight	Overweight
80-84	105	15.7 ± 3.8	14.8 ± 3.0	15.7 ± 4.4	16.8 ± 2.3	47	24.6 ± 6.1	22.9 ± 6.4	24.5 ± 5.2	27.3 ± 7.5
85-89	67	14.7 ± 4.2	14.1 ± 4.4	15.5 ± 3.5	14.1 ± 5.1	42	20.1 ± 5.0	21.6 ± 3.4	15.6 ± 5.2	20.4 ± 7.1
≥90	27	14.7 ± 5.5	13.1 ± 1.6	14.1 ± 5.9	12 ± 0.0	20	16.5 ± 4.5	16.0 ± 5.3	16.0 ± 4.8	19.2 ± 2.5

**Table 3:** Association between HGS and IADLs, ADL, risk of fall, and other factors on multiple regression model.

	Beta	*B*	95% CI *B*-coef	*p* value
Age	-0.196	-0.270	(-0.397)-(-0.143)	<0.001
Female (male)	-0.443	-5.361	(-6.594)-(-4.127)	<0.001
Illiterate (primary school and higher)	-0.130	-1.581	(-2.742)-(-0.419)	0.008
High school/higher (secondary or lower)	0.079	2.886	(-0.403)-6.175	0.085
Single/widowed (married)	-0.022	-0.264	-1.406-0.878	0.649
Number of current medications	0.005	0.041	-0.777-0.860	0.921
Risk of fall (TUG score)	-0.114	-1.328	(-2.400)-(0.255)	0.015
IADLs total score	0.153	0.344	0.134-0.554	0.001
ADL total score	0.044	0.595	-0.612-1.802	0.333

The result was present in variables (reference). Beta: standardized regression coefficient; *B*: unstandardized regression coefficient. The variables included in this model were chosen if *p* value ≤ 0.2 in Table 1. Activities of daily living (ADL) score (range 0–6, a higher number indicate higher independence). Instrumental activities of daily living scale (IADLs) score (range 0-8, a higher number indicate higher independence).

## Data Availability

The datasets of this study are available from the corresponding author on reasonable request.
